The article "Astragaloside IV controls collagen reduction in photoaging skin by improving transforming growth factor-β/Smad signaling suppression and inhibiting matrix metalloproteinase-1" was published in 2015. Journal: Mol Med Rep.

# Astragaloside IV controls collagen reduction in photoaging skin by improving transforming growth factor-β/Smad signaling suppression and inhibiting matrix metalloproteinase-1

**DOI:** 10.3892/mmr.2015.3212

**Published:** 2015-01-16

**Authors:** BIN CHEN, RAN LI, NING YAN, GANG CHEN, WEN QIAN, HUI-LI JIANG, CHAO JI, ZHI-GANG BI

**Affiliations:** 1 Department of Dermatology, The First Affiliated Hospital of Nanjing Medical University, Nanjing, Jiangsu 210024, P.R. China; 2 Department of Dermatology, The First Affiliated Hospital of Fujian Medical University, Fuzhou, Fujian 350005, P.R. China; 3 Department of Dermatology, BenQ Medical Center, Nanjing Medical University, Nanjing, Jiangsu 210019, P.R. China

**Keywords:** photoaging, astragaloside IV, type I procollagen, matrix metalloproteinase, transforming growth factor-β/Smad signaling

## Abstract

Exposure to ultraviolet (UV) light reduces levels of type I collagen in the dermis and results in human skin damage and premature skin aging (photoaging). This leads to a wrinkled appearance through the inhibition of transforming growth factor-β (TGF-β)/Smad signaling. UV irradiation increases type I collagen degradation through upregulating matrix metalloproteinase (MMP) expression. Astragaloside IV (AST) is one of the major active components extracted from *Astragalus membranaceus*. However, its multiple anti-photoaging effects remain to be elucidated. In the present study, the effects of AST against collagen reduction in UV-induced skin aging in human skin fibroblasts were investigated. The expression of type I procollagen (COL1), MMP-1, TGF-βRII and Smad7 were determined using reverse transcription-polymerase chain reaction, western blotting and ELISA, respectively. UV irradiation inhibits type I collagen production by suppressing the TGF-β/Smad signaling pathway and increasing COL1 degradation by inducing MMP-1 expression. Transforming growth factor-β type II protein and COL1 mRNA decreased but MMP-1 and Smad7 levels increased in the photoaging model group, which was reversed by topical application of AST. AST prevents collagen reduction from UV irradiation in photoaging skin by improving TGF-β/Smad signaling suppression and inhibiting MMP-1, thus AST may be a potential agent against skin photoaging.

## Introduction

Ultraviolet (UV) irradiation impairs human skin and causes premature skin aging (photoaging), which results in deep wrinkles and pigment formation (1,2). Type I collagen, the most abundant structural protein in skin connective tissue, is essential for maintaining the strength and elasticity of the skin. Disorganization, fragmentation and dispersion of collagen bundles are three characteristics in human photoaging skin (1,3). Destroying the structural integrity of the collagenous extracellular matrix is well-established to be the major reason for the wrinkled appearance of photoaged skin (4). UV irradiation decreases type I collagen through two interdependent pathways: Stimulation of collagen degradation and inhibition of type I procollagen (COL1) production (3,5). Thus, UV-induced control of type I collagen production is one of the critical factors in the mechanism of photoaging.

The article "Astragaloside IV controls collagen reduction in photoaging skin by improving transforming growth factor-β/Smad signaling suppression and inhibiting matrix metalloproteinase-1" was published in 2015. Journal: Mol Med Rep.

Transforming growth factor-β (TGF-β) is the primary regulator of collagen synthesis in human skin (6–9). TGF-β functions by binding to specific receptor complexes, including TGF-β type I (TβRI) and TGF-β type II (TβRII) receptors on the cell surface (9). Smad7 is one of the negative factors in the TGF-β/Smad signaling pathway, which interacts with TβRI to prevent activation of Smad2/3, thereby inhibiting TGF-β signaling. It has been reported that UV irradiation impairs TGF-β/Smad signaling through downregulating the transcription of TβRII. This impairment is a major reason for the reduced procollagen synthesis in human skin fibroblasts (10). For this reason, the prevention of UV-induced loss of TβRII may precede the recovery of type I collagen reduction in photoaging skin.

UV irradiation leads to direct or indirect DNA damage and the formation of radical oxygen species, which causes the subsequent activation of complex signaling pathways, followed by the induction of matrix metalloproteinases (MMPs) in skin cells. MMPs are a group of extracellular matrix (ECM) enzymes, which can degrade the protein components of the ECM (11). Upregulation of MMPs, particularly collagenase-1 (MMP-1), generated by several types of cells, including fibroblasts, keratinocytes, endothelial cells, macrophages, hepatocytes, chondrocytes and osteoblasts, is responsible for the lysis of dermal collagen in skin aging.

Astragaloside IV (AST) is a small molecular saponin with multiple activities under pathophysiological conditions, including antihypertensive, positive inotropic action, anti-inflammatory and anti-infarct properties. However, the effect of AST in photoaging skin remains to be elucidated. The present study focused on whether AST prevents collagen degradation in photoaging skin and the possible underlying mechanisms, *in vivo* and *in vitro* to determine whether AST inhibits collagen reduction in photoaging skin by improving TGF-β/Smad signaling suppression and inhibiting MMP-1.

## Materials and methods

### Chemicals and reagents

Rabbit polyclonal immunoglobulin G (IgG) anti-TβRII (sc-220) and mouse monoclonal IgG_2b_ anti-tubulin (sc-23950) antibodies were purchased from Santa Cruz Biotechnology, Inc. (Dallas, TX, USA).

The article "Astragaloside IV controls collagen reduction in photoaging skin by improving transforming growth factor-β/Smad signaling suppression and inhibiting matrix metalloproteinase-1" was published in 2015. Journal: Mol Med Rep.

### Cell culture

Human skin fibroblasts (HSFs), derived from newborn skin were acquired from the Chinese Academy of Medical Science (Beijing, China). The cells were then cultured in Dulbecco’s modified Eagle’s medium (DMEM; Hyclone, Logan, UT, USA), supplemented with 10% fetal calf serum (FCS; Invitrogen Life Technologies, Victoria, Australia), 100 U/ml penicillin and 100 μg/ml streptomycin (Sigma-Aldrich, St. Louis, MO, USA). HSFs were cultivated in 75-cm^2^ culture flasks in an incubator at 37°C with a humidified atmosphere containing 5% carbon dioxide. When the cells reached 80–90% confluency, they were subcultivated to 60-mm culture dishes.

### UVB irradiation

A total of four F36T12 ERE-VHO UV tubes were used in the present study as the UV source. A Kodacel TA401/407 filter (Kodak, Tokyo, Japan) was mounted 4 cm in front of the tubes to block UVC (wavelengths >290 nm). The irradiation intensity was monitored using a UVR radiometer equipped with a UVA sensor (Bioblock Scientific, Tournai, Belgium). Subconfluent HSFs were cultured in DMEM containing 0.1% FCS for 24 h and subsequently incubated in DMEM with various concentrations of AST (10, 20, 30, 40, 50 μml; Sigma-Aldrich) for 24 h. HSFs were then washed twice with fresh phosphate-buffered saline (PBS; Sigma-Aldrich) and exposed to UVA irradiation (10 J/cm^2^) in a thin layer of PBS. Following irradiation, the cells were incubated in DMEM for the indicated time.

### Western blotting

A total of 40 μg of protein from each sample was separated by 10–12% SDS-PAGE and transferred onto a polyvinylidene difluoride membrane (EMD Millipore, Bedford, MA, USA). Following blocking with 10% instant non-fat dry milk for 1 h, membranes were incubated with specific antibodies overnight at 4°C followed by incubation with horseradish-conjugated secondary IgG antibodies (anti-rabbit, #7074 and anti-mouse, #7076; Cell Signaling Technology, Inc., Danvers, MA, USA) for 1 h. Antibody binding was detected with the enhanced chemiluminescence detection system (Amersham Biosciences, Piscataway, NJ, USA).

### Cell viability assay

Cell viability was measured using the 3-(4,5-dimethylthylthiazol-2-yl)-2,5 diphenyltetrazolium bromide (MTT) method as described previously (12).

### Quantification of apoptosis by ELISA

The ELISA Detection kit (Roche, Palo Alto, CA, USA) was used to detect MMP-1 and Smad7 in HSFs with different treatments. Briefly, following the indicated treatments, the cytoplasmic histone/DNA fragments from cells were extracted and bound to immobilized anti-histone antibody. Subsequently, the peroxidase-conjugated anti-DNA antibody was used for the detection of immobilized histone/DNA fragments The antibodies used were from the ELISA Detection kit (Roche). Following the addition of a substrate for peroxidase, the spectrophotometric absorbance of the samples was determined using the Dynatech MR5000 plate reader at 405 nm (Dynatech Laboratories, Chantilly, VA, USA).

The article "Astragaloside IV controls collagen reduction in photoaging skin by improving transforming growth factor-β/Smad signaling suppression and inhibiting matrix metalloproteinase-1" was published in 2015. Journal: Mol Med Rep.

### RNA isolation, reverse transcription-polymerase chain reaction (RT-PCR)

Total RNA was isolated from human skin (Chinese Academy of Medical Science) using TRIzol reagent (Invitrogen Life Technologies, Shanghai, China) and reverse transcription was conducted on 2 μg RNA using the PrimeScript RT reagent kit (TaKaRa Bio Inc. Ohtsu, Japan) and standard RT-PCR primers for human COL1: Forward: 5′-CGC CAT CAA GGT CTA CTG C-3′ and reverse: 5′-GAA TCC ATC GGT CAT GCT CT-3′ and tubulin forward, 5′-ATCAGCAATGCCTCCTGCAC-3′ and reverse, 5′-CGTCAAAGGTGGAGGAGTGG-3′. Data were normalized to tubulin expression and the untreated group was set as one. The PCR was semi-quantitative and the cycling conditions were 50°C for 2 min, 95°C for 1 min and 40 cycles of amplification at 95°C for 15 sec, 60°C for 1 min, followed by 95°C for 15 sec, 60°C for 30 sec and 95°C for 15 sec.

### Statistical analysis

The values in the figures are expressed as the mean ± standard deviation. The figures in the present study were representative of >3 different experiments. Statistical analysis of the data between the control and treated groups was performed using SPSS software version 6.0 (SPSS, Inc., Chicago, IL, USA). P<0.05 was considered to indicate a statistically significant difference.

## Results

### Effect of AST on cell viability in HSFs

Initially, it was assessed whether AST affects cell viability in HSFs using an MTT assay. As shown in Fig. 1, at a low concentration (20 μg/ml), AST did not affect cell viability. AST at 30 μg/ml exhibited almost a 25% increase in cell viability. When the concentration was 40 μg/ml, AST had the most significant effect (~50%) on HSFs compared with the control. Subsequently, the effect of AST on cell viability in UVA-exposed HSFs was examined. The results revealed that UVA irradiation (10 J/cm^2^) exhibited marked cytotoxicity. AST (40 μg/ml) enhanced cell viability in HSFs irradiated with UVA (Fig. 2).

### Effect of AST on UVA-induced COL1 downregulation

Type I collagen is the most abundant structural protein in skin connective tissue. UV irradiation decreases type I collagen through inhibition of COL1 production. Therefore, the present study aimed to elucidate the effect of AST on UVA-induced COL1 downregulation. HSFs were pretreated with AST. Following UVA irradiation, secreted COL1 in the supernatants were harvested and identified using RT-PCR. As shown in Fig. 3, COL1 secretion was inhibited by UVA, while AST reversed this inhibitory effect. These results suggested that AST significantly prevented UV-induced reduction of COL1 mRNA expression.

The article "Astragaloside IV controls collagen reduction in photoaging skin by improving transforming growth factor-β/Smad signaling suppression and inhibiting matrix metalloproteinase-1" was published in 2015. Journal: Mol Med Rep.

### Effect of AST on UVA-induced MMP-1 expression

It is well-established that UV irradiation damages human skin cells and causes photoaging. UVA and UVB irradiation of dermal fibroblasts induced MMP-1 expression, which is implicated in the degradation of human skin matrix proteins, including collagen and other components of the ECM. In the present study, to investigate whether AST affects the expression of MMP-1 in UVA-irradiated HSFs, cultured fibroblasts were pretreated with AST followed by UVA irradiation. MMP-1 protein levels were determined using ELISA. As expected, the results revealed that UVA irradiation significantly enhanced MMP-1 expression. The ELISA results demonstrated that pretreatment with AST markedly inhibited UVB-induced MMP-1 expression compared with the UVA-irradiated group (Fig. 4).

### Inhibitory effect of AST on UVA-induced Smad7 expression

Smad7 is one of the negative factors in the TGF-β/Smad signaling pathway, which interacts with TβRI to prevent activation of Smad2/3, thereby inhibiting TGF-β signaling. It was subsequently investigated whether AST affects the expression of Smad7 in UVA-irradiated HSFs. Smad7 protein levels were determined using ELISA. The results demonstrated that UVA irradiation significantly enhanced Smad7 expression and the expression of Smad7 induced by UVB irradiation was significantly attenuated by AST (Fig. 5).

### Effect of AST on UVA-induced TβRII downregulation

Significant progress has been made towards understanding the molecular mechanisms underlying the UV-induced TGF-β/Smad signaling pathway. It is reported that UV irradiation impairs TGF-β/Smad signaling through transcriptional downregulation of TβRII (7). The effect of AST on UVA-induced TβRII downregulation was further investigated. The results revealed that attenuated TβRII expression induced by UVA irradiation was significantly inhibited by AST pretreatment (Fig. 6).

## Discussion

UV radiation causes premature skin aging, which is termed photoaging. It has been well-established that this complicated procedure is due to UV-induced collagen degradation through its effects on various signaling factors, including MMP-1 in the TGF-β/Smad signaling pathway.

TGF-β is a major regulator of procollagen production in human skin. TGF-β acts through its cell surface receptors to activate transcription factors Smad 2/3, which regulate TGF-β target gene expression (6–9). Considering that regulation of COL1 expression occurs via a complicated mechanism, which remains to be elucidated, multiple studies have indicated that transcriptional regulation has a major role in controlling its production (13,14). Transcription of the COL1 gene is directly regulated by TGF-β via a Smad3 binding element in its promoter (15). It was reported that UV irradiation impairs the TGF-β/Smad pathway by downregulating its type-II receptor and inducing Smad7 (11,16), and this impairment reduces procollagen synthesis in UV-irradiated human skin. Therefore, the UV-induced reduction of TβRII and UV-induced increase of Smad7 may provide novel insights for the molecular mechanisms of photoaging and suppression of UV-induced downregulation of TβRII and upregulation of Smad7, which may lead to the identification of novel approaches for the prevention of photoaging. The present data indicated that AST inhibits the downregulation of TβRII and the upregulation of Smad7, followed by suppression of the reduction of COL1 synthesis in the AST group, which revealed that the pathway and signaling factors regulated by AST were involved in its functions against photoaging.

The article "Astragaloside IV controls collagen reduction in photoaging skin by improving transforming growth factor-β/Smad signaling suppression and inhibiting matrix metalloproteinase-1" was published in 2015. Journal: Mol Med Rep.

UV irradiation is known to induce expression of MMP-1, −3 and −9 in human skin *in vivo,* and cultured human skin cells *in vitro* (17). UV-induced MMP-1 expression induces the cleavage of collagen fibers. Once collagen is cleaved by MMP-1, collagen degradation is further promoted by MMP-3 and −9. MMP-1, termed fibroblast-type or interstitial collagenase, is secreted by fibroblasts, keratinocytes and macrophages. MMP-1 degrades collagens type I, II and III and is hypothesized to have a pivotal role in the process of photoaging (18). These properties render MMP-1 an attractive target for the pharmacological development of anti-photoaging agents. Therefore, in the present study, the effect of AST on UV-induced MMP-1 expression was examined. It was identified that MMP-1 expression was significantly lower in the AST group. The results suggest that AST is a potent inhibitor of UV-induced MMP-1 expression.

In conclusion, the present findings demonstrated that AST inhibits UV-induced COL1 decrease by stimulating the TGF-β/Smad signaling pathway through upregulating TβRII and downregulating Smad7 as well as suppressing MMP-1 expression. Therefore, it is hypothesized that AST may be a potentially effective agent for the prevention of photoaging.

## Figures and Tables

**Figure 1:** Effect of AST on cell viability in human skin fibroblasts. Human fibroblasts were treated with or without AST for 24 h. The cytotoxicity was measured using an 3-(4,5-dimethylthylthiazol-2-yl)-2,5 diphenyltetrazolium bromide assay. Absorbance was read on a microplate reader at 490 nm. Results are expressed as the mean ± standard deviation of three independent experiments performed in triplicate. ^*^P<0.05 compared with the ctrl group. AST, astragaloside IV; OD, optical density; ctrl, control.

The article "Astragaloside IV controls collagen reduction in photoaging skin by improving transforming growth factor-β/Smad signaling suppression and inhibiting matrix metalloproteinase-1" was published in 2015. Journal: Mol Med Rep.

**Figure 2:** Effect of AST on cell viability in UV-exposed human skin fibroblasts. Fibroblasts were pretreated with indicated concentrations of AST for 24 h, followed by irradiation with UVA (10 J/cm^2^). The cells were then further cultured for 24 h. Cytotoxicity was measured using an 3-(4,5-dimethylthylthiazol-2-yl)-2,5 diphenyltetrazolium bromide assay. Absorbance was read on a microplate reader at 490 nm. Results are expressed as the mean ± standard deviation of three independent experiments performed in triplicate. ^**^P<0.05, compared with the ctrl group. ^#^P<0.05, compared with the UVA-irradiated only ctrl group. AST, astragaloside IV; OD, optical density; UV, ultraviolet; Ctrl, control.

**Figure 3:** Effect of AST on UVA-induced COL1 mRNA downregulation. Human skin fibroblasts were pretreated with the indicated concentrations of AST for 24 h, followed by irradiation with UVA (10 J/cm^2^) and then incubated for 24 h. Culture supernatants were harvested and COL1 mRNA expression was determined by reverse transcription-polymerase chain reaction. Results are expressed as the mean ± standard deviation of three independent experiments performed in triplicates. ^**^P<0.05, compared with the ctrl; ^*^P<0.05, compared with the UVA-irradiated only ctrlgroup. AST, astragaloside IV; UV, ultraviolet; Ctrl, control; COL1, type I procollagen.

**Figure 4:** Effect of AST on UVA-induced MMP-1 expression. Human skin fibroblasts were pretreated with the indicated concentrations of AST for 24 h, followed by irradiation with UVA (10 J/cm^2^), and then incubated for 24 h. Culture supernatants were harvested and MMP-1 protein in the supernatants was determined with an ELISA immunoassay kit. Results are expressed as the mean ± standard deviation of three independent experiments. ^*^P<0.05 compared with the ctrl, ^**^P<0.05, compared with the UVA-irradiated only ctrl group. AST, astragaloside IV; UV, ultraviolet; Ctrl, control; MMP-1, matrix metalloproteinase-1.

**Figure 5:** Effect of AST on UVA-induced Smad7 expression. Human skin fibroblasts were pretreated with the indicated concentrations of AST for 24 h, followed by irradiation with UVA (10 J/cm^2^), and then incubated for 24 h. The culture supernatants were harvested and Smad7 protein in the supernatants was determined with an ELISA immunoassay kit. Results are expressed as the mean ± standard deviation of three independent experiments. ^*^P<0.05 compared with the ctrl, ^**^P<0.05, compared with the UVA-irradiated only ctrl group. AST, astragaloside IV; UV, ultraviolet; Ctrl, control.

The article "Astragaloside IV controls collagen reduction in photoaging skin by improving transforming growth factor-β/Smad signaling suppression and inhibiting matrix metalloproteinase-1" was published in 2015. Journal: Mol Med Rep.

**Figure 6:** Effect of AST on UVA-induced TβR II downregulation. Human skin fibroblasts were pretreated with indicated concentrations of AST for 24 h, followed by irradiation with UVA (10 J/cm^2^) and then incubated for 24 h. Expression of TβRII was determined by western blotting. Results are expressed as the mean ± standard deviation of three independent experiments. ^**^P<0.05, compared with the ctrl. ^*^P<0.05, compared with the UVA-irradiated only ctrl group. AST, astragaloside IV; UV, ultraviolet; Ctrl, control; TβR II, transforming growth factor-β type II.
